# Deleterious Effects of Amoxicillin on Immune System and Haematobiochemical Parameters of a Rabbit

This article has been retracted.

**DOI:** 10.1155/2022/8691261

**Published:** 2022-03-23

**Authors:** Khalid Hussain, Mushtaq Hussain Lashari, Umer Farooq, Tahir Mehmood

**Affiliations:** ^1^Department of Zoology, The Islamia University of Bahawalpur, Bahawalpur, Pakistan; ^2^Department of Physiology, Faculty of Veterinary and Animal Sciences, The Islamia University of Bahawalpur, Pakistan; ^3^Centre for Applied Molecular Biology (CAMB), University of the Punjab, Lahore, 53700 Punjab, Pakistan

## Abstract

The present study is aimed at evaluating the haematobiochemical and immune system alterations in rabbit's exposure to amoxicillin. Thirty-two healthy rabbits were randomly divided into four (*n* = 8) groups comprising of three experimental groups and one control group. After 7 days of the acclimatization period, the study animals were given different doses of amoxicillin orally (100, 150, and 200 mg/kg body weight) for 21 days. The hematological results revealed that red blood cells, hemoglobin, mean corpuscular hemoglobin, and mean corpuscular hemoglobin concentration decreased significantly (*P* < 0.05) whereas white blood cells, neutrophils, and granulocyte exhibited a significantly increasing trend. Serum biochemical analysis showed a significantly increased concentration of HDL, LDL, serum globulin cholesterol, triglyceride, urea, uric acid, creatine, and calcium while plasma fibrinogen, blood sugar, albumin, and total protein were decreased significantly. Furthermore, liver function enzymes such as alanine transaminase (ALT), aspartate transaminase (AST), alkaline phosphatase (ALP), lactate dehydrogenase (LDH), and bilirubin significantly increased. Antioxidant enzymes and oxidative stress parameters such as malondialdehyde concentrations (MDA) increased significantly while catalase, superoxide dismutase, reduced glutathione, and peroxidase reduced significantly in antibiotic amoxicillin-treated groups as compared to the untreated control group (*P* < 0.05). Microscopic histopathological examination showed negative structural changes in liver, kidney, and heart tissues due to karyorrhexis; a disorganized hepatic cord in the liver; increased Bowman's space, necrotic renal tubules, and degenerative glomerulus in the kidney; and necrotic cardiac cells and cytoplasmic vacuolization in the heart, in antibiotic amoxicillin-treated rabbit groups as compared to the control group. In conclusion, amoxicillin induced stress and physiological and immunological impairments due to the adverse effects on haematobiochemical parameters and histopathological and tissue protein changes in target animals.

## 1. Introduction

Development in technology, industrial expansion, and extensive use of synthetic chemicals to enhance the production potential of crops and livestock animals and to control various diseases have become huge threats to both the environment and public health [1, 2]. Exposure to various environmental pollutants, industrial wastes, insecticide, pesticide, and heavy metals and the use of antibiotics in different animals and human not only induce death but also affect the life expectancy of various organisms [3]. Numerous studies highlighted that different synthetic compounds including antibiotics from multiple resources directly enter into public health ultimately leading to adverse effects [4]. Exposure to such type of antibiotics induces disturbance in normal physiological functions and reproductive dysfunction in target and nontarget animals [5]. Feeding to increasing human population is a global problem with thorough rethinking to increase food production especially from livestock to meet the global demand that can be mainly achieved through the prevention and treatment of stock from bacterial infections [6]. Antibiotics play a vital role in controlling pathogenic infections for a long time [7]. Tetracyclines, oxytetracyclines, sulfamethazine, penicillin G, and lincomycin are extensively used in veterinary practice to treat bacterial infections [8], although antibiotics are generally considered safe and well tolerated but still associated with a wide range of adverse effects. Multiple ranges of the pharmacodynamic effects of different antibiotics on blood constituents, serum enzymes, and electrolytes of the laboratory and domesticated animals are observed [9], including mutagenicity, nephropathy (gentamicin), hepatotoxicity, bone marrow toxicity, reproductive dysfunction (chloramphenicol), and carcinogenicity (oxytetracycline). The long-term antibiotic abuse leads to increase of drug-resistant bacteria for humans and animals. Amoxicillin is extensively used in the treatment of a wide range of diseases in veterinary and human. Amoxicillin is a bactericidal aminopenicillin, which eliminates principally by tubular secretion and glomerular filtration. Due to its broad spectrum activity, cheapness, favorable pharmacokinetics, and antimicrobial efficacy, amoxicillin is widely used in the poultry industry [10] and for preoperative antibiotic prophylaxis in veterinary medicine [11]. Since antibiotics are associated with adverse effects, the European Union introduced a general prohibition for the use of antibiotics as growth promoters [12]. Besides that, mostly, livestock producers use variable doses of various antibiotics to treat various kinds of infections in livestock. It is also a common practice to treat the entire stock, regardless of the affected ones [13]. Furthermore, antibiotics are also being recommended improperly for viral infections. These practices eventually lead to antibiotic remains entering the human food chain through an animal-derived food source such as meat, milk, and eggs and also become the reason of several health concerns in human beings along with livestock. But the mechanism of work about these antibiotics is still not clearly understood, and a lot of debates have been going on among scientists and researchers to conclude their adverse side effects. Therefore, the present study is designed to investigate the possible haematobiochemical and histopathological changes in a healthy local breed of rabbit after administration of variable doses of amoxicillin.

## 2. Materials and Methods

Apparently, 32 healthy adult rabbits (*Oryctolagus cuniculus*), about 1 year old (weight 1.5 kg), were collected from local market in Bahawalpur, Punjab. The study was approved in full by the “ethical review committee for the use of animals” which comes under the administrative control of the office of research, innovation and commercialization of the Islamia University of Bahawalpur, Pakistan. The rabbits were then transferred to a laboratory of animal toxicology in the department of zoology, the Islamia University of Bahawalpur, Pakistan. After that, rabbits were kept under similar management and environmental conditions, for example, the laboratory temperature was maintained at 25–27°C throughout the study. After shifting, rabbits were given the adjustment period to the research laboratory conditions for 7 days. During the adjustment period, drinking water was changed on a daily basis ad libitum and fed twice daily seasonal fodder *Trifolium alexandrinum* in the morning and evening. Rabbits were divided into 4 groups composed of 3 experimental and 1 control with 8 rabbits each group. Amoxicillin of GlaxoSmithKline was bought from a registered pharmaceutical shop in Bahawalpur. Variable doses of amoxicillin 100 mg/kg, 150 mg/kg, and 200 mg/kg body weight were fed orally to the animals of experimental groups A, B, and C, respectively, on a daily basis for 21 days, to investigate its effects on hematology and serum biochemistry.

### 2.1. Blood and Serum Analysis

Three mL of blood was collected from the marginal ear vein for hematological and biochemical analysis. Hematological parameters such as red blood cell count, hemoglobin, hematocrit, and total and differential white blood cell count were evaluated by using a hematological analyzer. The serum was used to estimate different liver function tests such as ALT and ALP which were determined according to earlier protocol plasma glucose concentrations, plasma urea concentrations, plasma creatinine, serum calcium, plasma albumin, total protein, cholesterol, and triglycerides, and uric acid was determined by using a Chem Analyzer model, BTS BioSystem, Spain, and diagnostic kits manufactured by BioMed Diagnostics, GmbH, Germany, following the user's manual.

### 2.2. Statistical Analysis

The data from all study groups were statistically analyzed by using Statistical Package for Social Sciences (SPPSS) and was expressed as mean ± SD. One-way ANOVA with Tukey's as a post hoc test was applied with a significance level set at *P* < 0.05.

## 3. Results

### 3.1. Clinical Signs

Clinical signs such as diarrhea, loss of body weight, tremors, skin coloration, lacrimation, gasping, dilation of pupil, and faintness were observed from mild to very severe in antibiotic amoxicillin-treated groups when compared with control groups (Table 1).

### 3.2. Relative Body and Organ Weight of Rabbits

Body weight of treated rabbits (groups) reduced significantly which were exposed to variable doses of amoxicillin as compared to that of the untreated control group. The relative weight of organs like the liver, kidney, heart, brain, and ovary decreased significantly whereas the relative weight of organs like the lungs, spleen, and testis increased significantly in the antibiotic amoxicillin-treated group as compared to the control group (Table 2).

### 3.3. Hematological Studies

The analysis of hematological parameters of control and experimental groups showed that total white blood cells (total WBC), granulocytes, neutrophils, and platelets significantly increased while red blood cells, hemoglobin, hematocrit, mean corpuscular volume (MCH), mean corpuscular hemoglobin concentration (MCHC), lymphocyte, and monocyte significantly decreased as compared to the control group. The values of the mean corpuscular volume (MCV) showed nonsignificant difference in antibiotic-treated groups as compared to the controlled group (*P* < 0.05) (Table 3).

### 3.4. Biochemical Parameter

The analysis of serum biochemical parameters of control and experimental groups showed that concentrations of HD lipoproteins, LD lipoproteins, cholesterol, triglyceride, urea, uric acid, creatine, calcium, and serum globulin significantly increased while blood sugar, albumin, total protein, and plasma fibrinogen significantly decreased in antibiotic-treated groups when compared to the controlled group (*P* < 0.05) (Table 4).

### 3.5. Antioxidant Enzymes

Analyses from the results of antioxidant enzymes and oxidative stress biomarker showed that values of malondialdehyde concentrations (MDA) increased significantly while catalase, superoxide dismutase, reduced glutathione, and peroxidase reduced significantly in antibiotic amoxicillin-treated groups as compared to the untreated control group (*P* < 0.05) (Table 5).

### 3.6. Liver Function Enzymes

Liver function tests showed that ALT, AST, ALP, LDH, and bilirubin of antibiotic-treated rabbits groups significantly increased as compared to those of the control group (*P* < 0.05) (Table 6).

### 3.7. Gross and Histopathological Studies

Histopathological examination of the liver showed karyorrhexis, cytoplasmic vacuolation, disorganized hepatic cord, bile duct hyperplasia, necrosis, and hydropic changes in hepatocytes. In the kidney, different pathological ailments like increased Bowman's space, congestion, necrosis of renal tubular epithelial cell, nuclear hypertrophy, necrosis of renal tubules, degeneration of the renal tubule, degenerative changes in kidney glomerulus, widening of the urinary space, hemorrhage b/w tubule, and cell infiltration with pyknotic nuclei were observed, while in heart necrosis of cardiac cells, cytoplasmic vacuolization, congestion, neutrophilic myocarditis, myofibrillolysis, and pyknotic nuclei in amoxicillin-treated rabbits were seen after 21 days of exposure to a higher dose (200 mg/kg body weight) of antibiotic amoxicillin-treated rabbit groups as compared to the control group (Table 7 and Figure 1).

## 4. Discussion

The results on the hematological profile exhibited an increased population of the total leukocytic count. The increased population of these cells in treated rabbits can be related to different tissue damages by amoxicillin. Different previous studies have also reported similar results in amoxicillin-treated sheep [11]. The present study showed that granulocytes significantly increased. This shows that amoxicillin treatment induced severe damage to the vital organ of rabbits; as a result, granulocytes increased to counter that damage. In present study, neutrophils significantly increased in experimental groups when compared with control ones and the increased number of neutrophils also shows that the damage is caused to blood-forming tissues in bone marrow along with other vital organs of the rabbits. In present study, lymphocyte significantly decreased in experimental groups as compared to the control group. Lymphocytopenia could be due to its decreased production of from bone marrow or its destruction in the body. In this study, monocyte significantly decreased in experimental groups as compared to the control group. Monocytopenia might be due to its decreased production of from bone marrow or its destruction in the body.

Similar findings were reported by Similar findings were reported by Olaniyan Added in list& Oladega, 2019, as increased blood platelets. This significant increase in platelet number shows that amoxicillin induced bleeding with organ and tissue damage; as a result, platelets increase to control bleeding or injury that occurs in the rabbit body. But a contrary result reported in platelets with a significantly decreasing trend was observed when the rabbits were given subcutaneous injection of amoxicillin supplemented with raw cucumber fruit juice (Olaniyan & Oladega, 2019).

In present study, red blood cells (RBC) significantly decreased in experimental groups as compared to the control group. Similar findings were observed by Added in list & Oladega, (2019). Contrary to our result of a significant decrease, a significantly increasing pattern was observed in RBC count when rabbits were supplemented with raw cucumber fruit juice (Olaniyan & Oladega, 2019).

In present study, hemoglobin (HB) significantly decreased in the experimental groups as compared to the control group. Similar results to those of ours were observed when the rabbits were given subcutaneous injection of amoxicillin supplemented with raw cucumber fruit juice. This could be as a result of the destruction of red blood cells or reduced production from haemopoietic tissues of the rabbit (Added in list & Oladega, 2019). As a result, a decreased concentration of hemoglobin is reported because hemoglobin is a constituent of RBC. Contrary to our result of a significant decrease, a significantly increasing trend was observed in hemoglobin concentration when rabbits were supplemented with raw cucumber fruit juice (Olaniyan & Oladega, 2019) (Table 3). This present study showed that hematocrit (HCT) significantly decreased in experimental groups as compared to the control group that is due to hemolysis of RBC; as a result, the number and size of RBC reduced that resulted in the reduction of hematocrit values.

The mean corpuscular volume (MCH) significantly decreased in experimental groups as compared to control. Destruction of RBC results in degradation of hemoglobin that results in a decreased average quantity of MCH in RBCs of rabbits. In present study, the mean corpuscular hemoglobin concentration (MCHC) significantly decreased in experimental groups as compared to the control group. Due to the adverse side effects of amoxicillin treatment, destruction of RBC occurred that results in degradation of hemoglobin as well as the decreased average quantity of MCHC blood of rabbits, while in our study, the mean corpuscular volume (MCV) means that the average size of red blood cells showed a nonsignificant difference in experimentally labelled groups.

During the current study, we observed a significantly increased trend of cholesterol in treated groups. Similar to the present result, a significant increase in cholesterol is also reported in sheep by Elmajdoub et al. In our study, we observed a significantly increasing trend in the triglyceride level of experimentally labeled groups.

The recent study showed a significantly increased urea level in experimental groups. Similar Added in list are reported in previous studies when subcutaneous injection of amoxicillin were given to rabbits (Olaniyan & Fowowe, 2020). This indicated nephrotoxicity as a result of overdose of amoxicillin which affects the kidneys, possibly causing poor kidney function (Olaniyan & Fowowe, 2020). In contrast to our results, a significant decrease in plasma urea was observed in rabbits following the administration of raw cucumber fruit juice supplementation (Olaniyan & Fowowe, 2020). In our study, the uric acid level significantly increased in antibiotic-treated groups because of kidney failure as a result of nephrotoxicity due to adverse side effects because of overdose treatment of amoxicillin to rabbits. In the present study, the creatine level significantly increased in treated groups due to renal failure that could be due to adverse side effects of amoxicillin on rabbits. Contrary to our result, a significant decrease in the creatinine level was revealed in the LZM-treated rabbit groups [14] (Table 4).

In the recent biochemical examination, we observed significantly increased concentrations of HD lipoproteins, LD lipoproteins, serum globulin, and calcium levels in antibiotic amoxicillin-treated groups with respect to the untreated control group. Similar to our results, increased concentrations of serum globulin are similar to LZM-fed rabbits [14]. In the present study, an increased concentration of high density lipoprotein is similar to another work in which Nigella sativa seed was fed to rabbits (16) A contrary to our result is reported by El-Deep et al. when they fed LZM to rabbits and found no significant difference. A contrary to our results of increased concentration of low-density lipoprotein is reported by El-Deep et al. when they fed LZM to rabbits and found no significant difference and also by El-Gindy et al. when they fed *Nigella sativa* seed as a diet to rabbits.

The present study showed that total protein, plasma fibrinogen, blood sugar, and albumin concentration significantly decreased in antibiotic-treated groups. Previously, in published literature, similar results of significantly decreased plasma albumin have also been reported in rabbits injected with amoxicillin supplemented with raw cucumber fruit juice. Hypoalbuminemia could be due to liver damage, hepatitis, and hepatotoxicity induced by amoxicillin because liver synthesizes albumin [16]. In contrast to our results, significantly increased plasma albumin is reported in rabbits supplemented with raw cucumber fruit juice [16].

The present results showed that malondialdehyde concentrations (MDA) increased significantly while reduced glutathione, catalase, superoxide dismutase, and peroxidase decreased significantly in antibiotic amoxicillin-treated groups as compared to the untreated control group. Our recent results of increased malondialdehyde concentration are contrary to those of El-Gindy et al. when they fed *Nigella sativa* seed to rabbits as compared to the basal diet-fed control group. Present results are also in contrary to those of Zweil et al. when they fed peppermint and basil essential oil as supplementation to evaluate productive performance of rabbits. A contrary to our result of MDA is reported by Imbabi et al. when they used fennel essential oil as an alternative for antibiotic. In the present study, we observed decreased catalase, reduced glutathione, superoxide dismutase, and peroxidase parameters and these results are in contrary with those of Singh et al. when they fed melon seed oil as dietary supplementation to rabbits and found a significant difference and no negative effect upon 0.6% on the antioxidant parameters such as superoxide dismutase (SOD), reduced glutathione (GSH), and malondialdehyde.

The serum ALT level and AST are commonly measured to determine hepatitis and hepatocellular injury possibly due to toxic substances such as drug and infectious agents as well as to estimate liver health (Olaniyan & Adepoju, 2019; [16]). In the current study, we found significantly increased levels of ALT, ALP, AST, LDH, and bilirubin in treated groups as compared to the untreated control group (Table 6). Previously, in published literature, similar results of a significant increase in ALT and AST values have also been reported in rabbits treated with amoxicillin supplemented with raw cucumber fruit juice. Increased plasma levels of ALT and AST can be caused by liver damage, hepatitis, and hepatotoxicity induced by amoxicillin. In contrast to our results, a significant decrease in plasma ALT and AST was observed in rabbits supplemented with raw cucumber fruit juice (Olaniyan & Adepoju, 2019). Furthermore, a significant decrease in the levels of ALT and AST was revealed by El-Deep et al. in LZM-treated rabbits. In our study, we investigated a significantly increased level of ALP in experimental-treated groups. Similar to our result, a significant increase in ALP is also reported in sheep by Elmajdoub et al. In our study, we observed that lactate dehydrogenase and bilirubin significantly increased in antibiotic-treated groups when compared with the control group.

Karyorrhexis, congestion of central vein, cytoplasmic vacuolation, disorganized hepatic cord, bile duct hyperplasia, necrosis and hydropic changes in hepatocytes, yknosis, vacuolar degeneration, hemorrhages, ceroid formation, nuclear hypertrophy, congestion, and degeneration of hepatocytes in liver were few indications of the present study, while previous studies reported that the amoxicillin-treated foetal liver showed vacuolar, fatty degenerations in the cytoplasm of the hepatocytes, devastations of mitochondria, and fragmentation of rough endoplasmic reticulum [17]. Previous studies also reported drug-induced liver injury, destruction of the biliary epithelium, lesions on the epithelium of interlobular ducts, and primary biliary cholangitis, such as inflammation and necrosis at the expense of cholangiocytes, bile duct loss, and biliary cirrhosis. Amoxicillin/clavulanic acid is associated with drug-induced liver injury and bile duct loss reported by the US Drug-Induced Liver Injury Network [18] [19] (Table 7). In our latest microscopic examination, we observed increased Bowman's space, congestion, necrosis of renal tubular epithelial cell, nuclear hypertrophy, necrosis of renal tubules, degeneration of renal tubule, degenerative changes in kidney glomerulus, widening of the urinary space, hemorrhage b/w tubule, and cell infiltration with pyknotic nuclei in the kidney of amoxicillin-treated rabbits, while previous studies reported that the renal cortex of maternally treated foetus showed erosion of the parietal cells of Bowman's capsule, hypoplasia of the mesangial cells of the glomerulus, and erosion of the epithelial cells lining the proximal and distal convoluted tubules. In the electron microscope level, the renal cortex of foetus maternally treated with amoxicillin showed fusion of the foot processes of the podocytes, partial destruction of the apical brush borders microvilli of the proximal convoluted tubule cells, degeneration of some mitochondria, and fragmentation of the rough endoplasmic reticulum elements [20] (Table 7). In recent microscopy, we observed necrosis of cardiac cells, cytoplasmic vacuolization, congestion, neutrophilic myocarditis, myofibrillolysis, and pyknotic nuclei in amoxicillin-treated rabbits, while in a previous study, no authentic and related research data are available on heart pathology in connection to our study (Table 7).

In conclusion, the results of the present study showed that amoxicillin administration at higher levels resulted in many adverse effects like haematobiochemical alterations, metabolism dysfunction, and suppressed immunity. Therefore, monitoring of this chemical is crucial to reduce the ill effects in public health.

## Figures and Tables

**Figure 1:** Photomicrograph of the liver (a); kidney (b), and heart (c) of treated rabbits (200 mg/kg body weight) showing different histopathological changes (400x, H&E stain).

**Table 1:** Severity of different clinical signs in rabbits exposed to variable doses of amoxicillin.

Clinical ailments	Groups/treatments			
	Control (0.0 mg/kg)	A (100 mg/kg)	B (150 mg/kg)	C (200 mg/kg)
Diarrhea	−	+	++	++++
Loss of body weight	−	+	+	+++
Tremors	−	+	++	+++
Gasping	−	++	+++	++++
Skin coloration	−	−	+++	+++
Lacrimation	−	+	+	++
Faintness	−	−	+++	++++
Dilation of pupil	−	−	+	++

Normal: −; mild: +; moderate: ++; severe: +++; very severe: ++++.

**Table 2:** Relative body and organ weight in rabbits injected with variable doses of amoxicillin.

Body and organ weight	Groups/treatments			
	Control (0.0 mg/kg)	A (100 mg/kg)	B (150 mg/kg)	C (200 mg/kg)
Body weight (g)	1289.3 ± 21.2	1223.5 ± 17.1^∗^	1170.1 ± 10.4^∗^	1125.4 ± 5.3^∗^
Liver (×10^3^ ppm)	33.95 ± 0.31	31.40 ± 1.54^∗^	29.50 ± 0.51^∗^	27.70 ± 1.30^∗^
Kidney (×10^3^ ppm)	4.78 ± 0.36	3.33 ± 0.60^∗^	3.19 ± 0.18^∗^	2.97 ± 0.13^∗^
Lungs (×10^3^ ppm)	5.62 ± 0.13	7.18 ± 5.63^∗^	7.71 ± 0.44^∗^	8.66 ± 0.69^∗^
Heart (×10^3^ ppm)	3.90 ± 0.20	2.79 ± 0.34^∗^	2.47 ± 0.04^∗^	2.22 ± 0.13^∗^
Brain (×10^3^ ppm)	6.91 ± 0.29	5.73 ± 1.10^∗^	4.8 ± 0.21^∗^	4.22 ± 0.43^∗^
Spleen (×10^3^ ppm)	281.00 ± 52.70	298.00 ± 27.10^∗^	364.00 ± 28.30^∗^	398.00 ± 10.18^∗^
Testis (×10^3^ ppm)	828 ± 49.21	916 ± 24.51^∗^	952 ± 28.51^∗^	1080 ± 20.2^∗^
Ovary (×10^3^ ppm)	163.57 ± 6.51	161.23 ± 5.43^∗^	157.13 ± 2.66^∗^	146.23 ± 2.37^∗^

The data are represented as mean ± SD. Values bearing an asterisk in each row show significant difference as compared to that control group (*P* < 0.05).

**Table 3:** Hematological parameters of rabbits exposed to variable doses of amoxicillin.

Parameters	Groups/treatments			
	Control (0.0 mg/kg)	A (100 mg/kg)	B (150 mg/kg)	C (200 mg/kg)
Total white blood cells (10^3^/*μ*L)	4.96 ± 0.73	5.03 ± 0.63	6.46 ± 1.36^∗^	7.71 ± 1.26^∗^
Lymphocytes (10^3^/*μ*L)	3.77 ± 0.82	2.91 ± 0.58	2.53 ± 0.47^∗^	1.51 ± 0.28^∗^
Neutrophils (10^3^/*μ*L)	1.84 ± 0.88	2.18 ± 0.66	2.56 ± 0.48^∗^	3.82 ± 2.96^∗^
Monocytes (10^3^/*μ*L)	0.48 ± 0.12	0.40 ± 0.15	0.32 ± 0.13	0.21 ± 0.09^∗^
Granulocytes (10^3^/*μ*L)	2.21 ± 0.55	3.03 ± 0.45	3.23 ± 1.03^∗^	3.61 ± 0.73^∗^
Red blood cells (10^6^/*μ*L)	5.53 ± 0.90	5.52 ± 0.42	5.48 ± 0.50	4.36 ± 0.62^∗^
Hemoglobin (g/dL)	11.46 ± 0.79	11.43 ± 1.91	10.93 ± 0.99	10.18 ± 1.47^∗^
Hematocrit (%)	38.05 ± 3.88	34.53 ± 5.73^∗^	34.26 ± 2.63^∗^	27.41 ± 3.80^∗^
Mean corpuscular volume (fL)	62.90 ± 1.88	68.87 ± 3.48^∗^	62.55 ± 2.59	62.35 ± 1.49
Mean corpuscular hemoglobin (pg)	23.36 ± 1.11	19.80 ± 0.74^∗^	20.93 ± 0.93^∗^	20.61 ± 0.74^∗^
Mean corpuscular hemoglobin concentration (g/dL)	37.13 ± 1.02	28.77 ± 0.63^∗^	33.46 ± 0.69^∗^	33.11 ± 0.51^∗^
Platelets (10^3^/*μ*L)	248.87 ± 38.65	291.50 ± 75.72^∗^	355.12 ± 87.64^∗^	430.12 ± 40.24^∗^

The data are represented as mean ± SD. Values bearing an asterisk in each row show significant difference as compared to the control group (*P* < 0.05).

**Table 4:** The biochemical parameters of rabbits exposed to variable doses of amoxicillin.

Parameters	Groups/treatments			
	Control (0.0 mg/kg)	A (100 mg/kg)	B (150 mg/kg)	C (200 mg/kg)
Blood sugar	111.37 ± 2.66	106.00 ± 3.02^∗^	105.25 ± 2.49^∗^	104.37 ± 1.68^∗^
Cholesterol	120.62 ± 3.88	124.25 ± 2.81^∗^	132.00 ± 4.34^∗^	137.00 ± 1.85^∗^
Triglyceride	144.62 ± 10.33	147.87 ± 3.90^∗^	158.25 ± 5.62^∗^	165.75 ± 7.42^∗^
Uric acid	1.93 ± 0.29	1.96 ± 0.25	2.20 ± 0.25^∗^	2.35 ± 0.20^∗^
Urea	36.25 ± 2.12	37.00 ± 2.13	38.12 ± 2.03^∗^	39.75 ± 2.05
Creatine	0.75 ± 0.14	0.80 ± 0.13	1.10 ± 0.20^∗^	1.27 ± 0.12^∗^
Calcium	10.71 ± 0.40	11.63 ± 0.44	11.72 ± 0.94^∗^	11.93 ± 0.77^∗^
Albumin	4.78 ± 0.18	4.37 ± 0.14	4.10 ± 0.13^∗^	3.85 ± 0.19^∗^
Total protein	6.66 ± 0.43	6.53 ± 0.21	6.01 ± 0.20^∗^	5.71 ± 0.29^∗^
HD lipoprotein (mg/dl)	41.33 ± 1.76	47.10 ± 2.90^∗^	57.03 ± 3.14^∗^	74.10 ± 4.10^∗^
LD lipoprotein (mg/dl)	14.10 ± 1.12	17.12 ± 1.77	26.80 ± 1.51^∗^	33.14 ± 1.65^∗^
Plasma fibrinogen	610.1 ± 303.7	464.7 ± 235.7^∗^	363.2 ± 65.2^∗^	290.0 ± 157.2^∗^
Serum globulins	2.31 ± 0.13	2.6 ± 0.11^∗^	2.80 ± 0.36^∗^	2.98 ± 0.23^∗^

The data are represented as mean ± SD. Values bearing an asterisk in each row show significant difference as compared to the control group (*P* < 0.05).

**Table 5:** Comparison of antioxidant enzymes of rabbits exposed to variable doses of amoxicillin.

Parameters	Groups/treatments			
	Control (0.0 mg/kg)	A (100 mg/kg)	B (150 mg/kg)	C (200 mg/kg)
Malondialdehyde concentrations	27.19 ± 1.12	28.15 ± 1.31	37.13 ± 3.23^∗^	52.67 ± 2.43^∗^
Catalase (U/mg p)	26.32 ± 3.50	23.32 ± 2.90^∗^	17.13 ± 1.10^∗^	13.12 ± 1.70^∗^
Superoxide dismutase (U/mg p)	32.16 ± 1.13	28.62 ± 1.80^∗^	22.80 ± 1.15^∗^	14.11 ± 1.13^∗^
Reduced glutathione (U/mg p)	31.70 ± 3.14	28.63 ± 2.19^∗^	22.92 ± 4.19^∗^	17.24 ± 2.13^∗^
Peroxidase (U/mg p)	2.51 ± 0.32	2.30 ± 0.21	1.62 ± 0.65^∗^	1.12 ± 0.11^∗^

The data are represented as mean ± SD. Values bearing an asterisk in each row show significant difference as compared to the control group (*P* < 0.05).

**Table 6:** Effect of variable doses of amoxicillin on liver function enzymes in rabbits.

Parameters	Groups			
	Control (0.0 mg/kg)	A (100 mg/kg)	B (150 mg/kg)	C (200 mg/kg)
Alanine aminotransferase (IU)	123.75 ± 4.80	132.37 ± 4.13^∗^	136.00 ± 3.02^∗^	140.25 ± 3.61^∗^
Alkaline phosphatase (IU)	227.75 ± 8.82	241.75 ± 6.75^∗^	249.12 ± 9.43^∗^	264.12 ± 4.79^∗^
Bilirubin (mg/dL)	0.52 ± 0.03	0.57 ± 0.01^∗^	0.61 ± 0.01^∗^	0.67 ± 0.02^∗^
Aspartate transaminase (IU)	106.00 ± 11.30	137.00 ± 28.30^∗^	159.50 ± 20.50^∗^	197.50 ± 21.90^∗^
Lactate dehydrogenase (IU)	445.70 ± 30.50	515.70 ± 218.50^∗^	664.70 ± 383.50^∗^	786.30 ± 364.90^∗^

The data are represented as mean ± SD. Values bearing an asterisk in each row show significant difference as compared to the control group (*P* < 0.05).

**Table 7:** Severity of different histopathological changes in organs of rabbits exposed to variable doses of amoxicillin.

Histopathological lesions	Groups/treatments		
	A (100 mg/kg)	B (150 mg/kg)	C (200 mg/kg)
Liver			
Karyorrhexis	+	++	++++
Congestion of central vein	−	−	+++
Cytoplasmic vacuolation	++	+++	++++
Disorganized hepatic cord	−	++	+++
Bile duct hyperplasia	+	+	+++
Necrosis and hydropic changes in hepatocytes	+	+++	+++
Pyknosis	+	++	++++
Vacuolar degeneration	++	++++	++++
Hemorrhages	+	++	+++
Ceroid formation	++	++	+++
Nuclear hypertrophy	++	++	++++
Congestion	++	+++	+++
Degeneration of hepatocyte	++	+++	++++

Kidney			
Increased Bowman's space	+	++	++++
Congestion	+	++	+++
Necrosis of renal tubular epithelial cell	+	++++	++++
Nuclear hypertrophy	+	+++	++++
Necrosis of renal tubules	+	+++	+++
Degeneration of renal tubule	+	+++	+++
Degenerative changes in kidney glomerulus	+	++	+++
Widening urinary space	+	+++	+++
Hemorrhage b/w tubule	+	+	++
Cell infiltration with pyknotic nuclei	+	++	+++

Heart			
Necrosis of cardiac cells	+	+++	++++
Cytoplasmic vacuolization	++	+++	++++
Congestion	+	+++	++++
Neutrophilic myocarditis	+	+++	++++
Myofibrillolysis	+	+++	++++
Pyknotic nuclei	+	++	+++

Normal: −; mild: +; moderate: ++; severe: +++; very severe: ++++.

## Data Availability

Data is openly available for readers.
